This article has been retracted.

# The Relationship between Ultrasonographic Features of Hepatocellular Carcinoma and the Severity of Hepatocellular Carcinoma and the Expression of PTEN and Tg737

**DOI:** 10.1155/2022/2608633

**Published:** 2022-03-24

**Authors:** Lei Tang, Yan Zhang, Qiong Zhou, Qiaojun Hong, Zhanggui Wang

**Affiliations:** ^1^Department of Oncology, Anhui No. 2 Provincial People's Hospital, Hefei 230041, China; ^2^Department of Radiotherapy, Anhui No. 2 Provincial People's Hospital, Hefei 230041, China

## Abstract

To investigate the relationship between the ultrasonographic features of hepatocellular carcinoma (HCC) and the severity of HCC and the expression of tumor suppressor genes PTEN and Tg737, 90 patients with primary liver cancer are selected as the study subjects. The enhancement of liver tumor in arterial phase, portal venous phase, and delayed phase is observed by contrast-enhanced ultrasound (CEUS) before operation, and the echo intensity is compared with that of surrounding liver parenchyma. Immunohistochemistry is used to detect the expression of PTEN and Tg737 in hepatocellular carcinoma and paracancerous tissues. (1) In HCC, CEUS enhancement is characterized by rapid enhancement in arterial phase, enhancement in portal venous phase and delayed phase, and decreased hypoechoic changes. About 78.0% of the stage I-II liver cancer and 85.0% of the stage III-IV liver cancer show rapid enhancement and high echo in the arterial phase; only 8.0% of the stage I-II liver cancer shows moderate echo changes in the portal venous phase, while 32.5% (13/40) stage III-IV liver cancer shows moderate echo changes in the portal venous phase. (2) The positive rates of PTEN in liver cancer tissues and paracancerous tissues are 21.1% (19/90) and 70.0% (63/90), respectively, and the difference is statistically significant. The positive rates of Tg737 in liver cancer tissues and paracancerous tissues are 17.8% (16/90) and 75.6% (68/90), respectively, and the difference is statistically significant. Compared with PTEN and Tg737 negative groups, the ascending slope (RS) and initial elimination time (WT) of PTEN and Tg737 positive groups are significantly higher, indicating that the inflow velocity of contrast medium in the positive group is higher, the outflow time is shorter, and the lesions shows low enhancement rapidly. However, the expression of PTEN and Tg737 had no significant difference in maximal intensity (IMAX), peak time (TTP), and mean transit time (mTT). (3) Correlation analysis shows that the immunohistochemical scores of PTEN and Tg737 are not significantly correlated with IMAX, mTT, and TTP but positively correlated with RS (*r* = 0.359,*P* < 0.05), suggesting that the positive expressions of PTEN and Tg737 are negatively correlated with the inflow velocity of contrast medium. The immunohistochemical scores of PTEN and Tg737 are negatively correlated with WT, which indicated that the higher the expression intensity of PTEN is, the longer the outflow time of contrast medium is and the slower the outflow of contrast medium is. There is a significant correlation between the expression of PTEN and Tg737 proteins and CEUS parameters in hepatocellular carcinoma.

## 1. Introduction

Liver cancer is one of the most common malignant tumors in China, with a high incidence in the southeast coastal areas. The median age of patients with liver cancer in China is 40 to 50 years old, and males are more common than females [1]. Its incidence has had an increasing trend in recent years. In China, the annual mortality rate of liver cancer accounts for the second place of cancer mortality and ranks the third among malignant tumors of digestive system, next to stomach and esophageal cancers. Hepatitis B, hepatitis C, liver cirrhosis, and hepatocyte necrosis are prone to malignant changes in the process of hepatocyte regeneration. Various carcinogens such as aflatoxin B2, organic carcinogens, chemicals, and algal toxins can also cause cancer [2].

At present, in addition to histopathological examination which is the only gold standard for the diagnosis of liver cancer, imaging examination has become one of the important standards. Conventional ultrasound or CT examination is the first choice for the diagnosis of liver cancer, but its specificity and sensitivity are low [3]. With the development of imaging technology, the application of contract enhanced ultrasound (CEUS) and enhanced CT/MRI in the qualitative diagnosis of liver cancer is becoming more and more mature [4]. CEUS technology has become more and more mature in the clinical diagnosis of many diseases. At the same time, interventional ultrasound is also widely used in clinic. The close combination of the two can find new advantages in clinical diagnosis and guiding treatment [5]. At present, CEUS has been successfully used in the evaluation of ultrasound-guided catheterization or interventional therapy, which can not be ignored in clinical diagnosis and treatment, especially in diagnosing the etiology of bile duct and urinary system obstruction and guiding ultrasound-guided minimally invasive interventional therapy [6]. At the same time, with the development and progress of medicine, the treatment of liver tumor has developed from single surgical resection to interventional therapy (microwave ablation, radiofrequency ablation, anhydrous alcohol injection, etc.) and palliative treatment [7]. For different sizes of tumor lesions, it is necessary to take into account the patient's own condition.

Only a better understanding of the differences between different imaging methods in diagnosing the size of different lesions and a more accurate measurement of lesion size can guide the selection of more appropriate treatment options prior to clinical procedures. PTEN is a recognized tumor suppressor gene located in 10q23.3, which can inhibit cell proliferation by blocking the cell cycle [8]. Its abnormal expression is also an important factor in tumor occurrence, development, invasion, and metastasis. Tg737 gene is distributed on the long arm of chromosome 13 and participates in the regulation of cell function, but its biological effect has not been fully understood at this stage. Previous studies have confirmed the abnormal expression of PTEN and Tg737 in HCC, but there are few studies on the relationship between their abnormal expression and ultrasonic parameters of HCC [9]. Therefore, the purpose of this study was to explore the correlation between the characteristics of CEUS, pathological parameters, and the expression of PTEN and Tg737 in patients with hepatocellular carcinoma (HCC).

## 2. The Proposed Method

### 2.1. The Object of Study

A total of 90 patients with primary liver cancer from January 2017 to June 2020 are selected for the study. Inclusion criteria are as follows: (1) all patients are diagnosed with hepatocellular carcinoma by cytological or pathological diagnosis. (2) All patients are diagnosed for the first time. (3) All patients are treated by operation, and the cancer tissues and paracancerous tissues are preserved in the laboratory or pathology department of our hospital. (4) Routine ultrasound and liver CEUS examination are performed before operation. Other diseases that may affect the results of liver CEUS examination are excluded. Among the 90 patients, there are 53 males and 37 females, with an average age of (63.8 ± 12.4) years. There are 79 cases of hepatitis B cirrhosis, 3 cases of hepatitis C cirrhosis, 2 cases of hepatitis B complicated with hepatitis C, 55 cases of right hepatectomy, 12 cases of middle lobectomy, 17 cases of left hepatectomy, and 6 cases of right hepatectomy.

### 2.2. Ultrasonic Examination

Logiq9/e9 color Doppler ultrasound diagnostic instrument (made by GE company in the United States) was used for testing. The probe frequency was 6–8 MHz and the contrast medium was SonoVue (produced by Bracco company in Italy). A routine plain scan was performed to determine the two-dimensional imaging parameters such as the scope, size, boundary, and number of lesions. At the same time, color Doppler imaging was superimposed on the basis of two-dimensional imaging to evaluate the echo of HCC, internal blood flow and its relationship with surrounding tissue structure, and the characteristics of internal enhancement and regression of HCC during contrast-enhanced ultrasound. The enhancement of liver tumor in arterial phase, portal venous phase, and delayed phase was observed and compared with that of surrounding liver parenchyma. The quantitative analysis of CEUS dynamic image data is carried out by using the SonoLiverCAP software developed by TomTec company, and the time-intensity curve is generated. CEUS parameters include the following indicators: RiseTime: from 10% to 90% of IMAX. Time to peak off (t) (TTP): the time from the beginning of the contrast medium to IMAX. Mean transit time corresponding to the center of gravity of f(t) (mTT): the time from the beginning to the decline of TIC to half of IMAX. Rise slope (RS): calculated according to the formula RS = IMAX/TTP. Start-up time (WT): the transition time of the contrast medium from IMAX to equivalent enhancement.

### 2.3. Immunohistochemical Detection of PTEN and Tg737 Expression

The paraffin sections are dewaxed with xylene, dehydrated by gradient concentration ethanol, and recovered by microwave sodium citrate buffer. PBS was added as a negative control, and anti-PTEN antibody and anti-Tg737 antibody are incubated at 4°C for the night. On the second day, the tissue was washed with PBS for 3 times and incubated with a ready-to-use universal mouse second antibody for 2 hours. The immunohistochemical score was scored by the semiquantitative method, and the staining intensity was divided into 3 grades: score 0 (no staining), score 1 (weak staining), and score 2 (strong staining). The area of positive cells was expressed as a percentage, score 0 (<25%), score 1 (25%–50%), score 2 (51%–75%), and score 3 (>75%), and the immunohistochemical score was calculated according to the formula: total score = positive area value × intensity score. The score ≥3 was judged as a positive expression.

### 2.4. Statistical Analysis

All data are analyzed by SPSS 20.0 software. The counting data are expressed by frequency, chi-square test was used, mean ± standard deviation was used for measurement data, and *t*-test was used for comparison between groups. *P* < 0.05 was considered that the difference was statistically significant.

## 3. Experimental Results

### 3.1. Ultrasonographic Features of Hepatocellular Carcinoma

CEUS examination of normal liver shows that the enhancement phase of hepatic artery began about 10–20 seconds after injection and lasted about 10–15 seconds, while the portal venous phase began after the arterial phase, about 30–45 seconds after injection, lasting about 2 min. Delayed imaging began after the portal vein phase and lasted for up to 6 min after injection. In HCC, CEUS enhancement was characterized by rapid enhancement in arterial phase, enhancement in portal venous phase and delayed phase, and decreased hypoechoic changes.  Figure 1 shows the ultrasonographic characteristics of liver cancer.

### 3.2. Correlation between Ultrasonographic Features and Pathological Staging of HCC

Ultrasonography shows rapid enhancement and hyperecho in stage I-II liver cancer of 78.0% (39/50) and hyperechoic in stage III-IV liver cancer of 85.0% (34/40), while that of stage I-II liver cancer shows rapid enhancement and hyperecho in arterial phase. About 8.0% of stage I-II HCC shows moderate echo changes in the portal venous phase, while the rest shows hypoechoic changes after extinction. About 32.5% (13/40) of stage III-IV liver cancer shows moderate echo changes in the portal venous phase. About 92.0% (46/50) of stage I-II liver cancer and 90.0% (36/40) of stage III-IV liver cancer show hypoechoic changes in the delayed phase. The results show that the liver cancer of stage I-II shows moderate echo changes in the portal venous phase, while the rest of the liver cancer shows hypoechoic changes in the portal venous phase. Stage I-II liver cancer shows moderate echo changes in the portal vein phase.  Table 1 lists the correlation between ultrasound characteristics and pathological stage.

### 3.3. Expression of PTEN and Tg737 Protein Detected by Western Blot

Western blot detection shows that the relative expressions of PTEN protein in cancer tissue and paracancerous tissue are (2.16 ± 0.23) and (0.76 ± 0.11). The expressions of Tg737 protein in cancer tissue and paracancerous tissue are (1.69 ± 0.16) and (0.68 ± 0.09), respectively, and the difference was statistically significant (*P* < 0.05). The results show that the relative expression of PTEN and Tg737 protein in paracancerous tissues of HCC was significantly higher than that in cancerous tissues.  Figure 2 shows the western blot analysis for the expression of PTEN and Tg737 protein.

### 3.4. Immunohistochemical Detection of PTEN Protein in Tissues

Immunohistochemical examination shows that the positive rate of PTEN in liver cancer tissue and paracancerous tissue was 21.1% (19/90) and 70.0% (63/90), respectively, and the difference was statistically significant (*χ*^2^ = 43.365, *P* = 0.000). In cancer cells, PTEN protein was obviously expressed in both cytoplasm and nucleus, while PTEN protein was mainly expressed in cytoplasm in paracancerous tissues.  Figure 3 shows the immunohistochemical detection of PTEN protein in tissues.

### 3.5. Immunohistochemical Detection of Tg737 Protein in Tissues

Immunohistochemical examination shows that the positive rate of Tg737 in liver cancer tissue and paracancerous tissue was 17.8% (16/90) and 75.6% (68/90), respectively, and the difference was statistically significant (*χ*^2^ = 53.689, *P*  = 0.000). In cancer tissues and paracancerous tissues, Tg737 protein was mainly expressed in the cytoplasm.  Figure 4 displays the immunohistochemical detection of Tg737 protein in tissues.

### 3.6. Effect of PTEN and Tg737 Expression on CEUS Parameters

CEUS parameters show that RS and WT in PTEN positive group are significantly higher than those in PTEN negative group, indicating that the inflow velocity of contrast medium in PTEN positive group is higher and the outflow time was shorter, and the lesions show low enhancement rapidly. However, there is no significant difference in the expression of PTEN on IMAX, TTP, and mTT. The effect of Tg737 expression on CEUS parameters is the same as that of PTEN.  Table 2 lists the effects of PTEN expression on the CEUS parameters.

### 3.7. Correlation between PTEN and Tg737 Expression and CEUS Parameters

There are 34 cases, 26 cases, 11 cases, 11 cases, 6 cases, and 2 cases of patients with PTEN immunohistochemical scores of 0, 1, 2, 3, 4, and 6, respectively. There are 35 cases, 28 cases, 11 cases, 9 cases, 6 cases, and 1 case with Tg737 immunohistochemical scores of 0, 1, 2, 3, 4, and 6, respectively. Correlation analysis shows that the immunohistochemical scores of PTEN and Tg737 are not significantly correlated with IMAX, mTT, and TTP, but they are significantly positively correlated with RS. The positive expression of PTEN and Tg737 was negatively correlated with the inflow velocity of contrast medium. The correlation analysis shows that the immunohistochemical scores of PTEN and Tg737 are positively correlated with the inflow velocity of contrast medium (*r* = 0.359, *P* < 0.05). The immunohistochemical scores of PTEN and Tg737 are negatively correlated with WT (*P* < 0.05), which indicated that the higher the expression intensity of PTEN and Tg737, the longer the outflow time of contrast medium and the slower the regression.  Figure 5 shows correlation analysis of immunohistochemical scores of PTEN, Tg737, and RS.

### 3.8. Influence of the Expression of PTEN and Tg737 on the Prognosis of Patients

Kaplan–Meier survival curve analysis shows that the 1-year overall survival rates of patients in the PTEN positive group and negative group are 40.0% (16/40) and 56.0% (28/50), respectively, and those in the Tg737 positive group and negative group are 25.0% (10/40) and 48.0% (24/50), respectively. The 1-year overall survival rate of patients in PTEN (*χ*^2^ = 2.634, *P* = 0.032) and Tg737 positive (*χ*^2^ = 1.982, *P* = 0.045) groups are significantly lower than that of their negative group.  Figure 6 shows the effects of PTEN and Tg737 expression on patient prognosis.

## 4. Clinical Data Analysis

Ultrasound diagnosis is a common and effective method to diagnose liver cancer. It is a non-invasive localization method with the advantages of low price, repeatability, no radiation damage, and high sensitivity. However, there are blind areas, which are difficult to detect, which are not only affected by the background of other liver diseases but also by the performance of the equipment and the anatomical knowledge and experience and operation of the operator [10]. The process of abundant blood supply and angiogenesis in the focus of liver cancer is exuberant, and a large number of neovascularization can provide nutrients for the growth of tumor cells. The malignant degree of liver cancer is high and the prognosis is poor, and the recurrence rate and mortality rate are high after treatment [11]. In clinical practice, accurate evaluation of the blood supply of liver cancer lesions can not only provide a basis for judging the severity of the disease but also provide a reference for the choice of treatment. Contrast-enhanced ultrasound is a method of ultrasound examination developed in recent years. The ultrasound contrast agent used is a kind of micron pure blood pool contrast agent, which can well reflect the local blood flow of the tissue. The blood flow characteristics are then assessed by quantitative parameters. In this study, the CEUS parameters of patients with hepatocellular carcinoma are analyzed [12]. The results show that the initial growth time, peak time, and peak acceleration time of the focus are less than those of the surrounding background liver tissue, and the initial enhancement rate and enhancement rate of the lesion are higher than those of the surrounding background liver tissue, which indicated that the number of neovascularization in the liver cancer tissue was larger, the vascular diameter was thicker, the resistance was lower, and the contrast medium entered the blood vessels faster [13].

Early hepatocellular carcinoma (HCC) usually has more arterial blood supply and less portal vein blood supply than the surrounding liver parenchyma. For all the vascular phases of ultrasound contrast agents, the multistep changes of the blood flow of these arteries and portal veins are the key factors in the differential diagnosis of hepatocellular carcinoma in the context of liver cirrhosis. In addition to the blood flow changes of the nodules, the evolution of HCC also shows an increase in the size of the nodules. With the increase of the diameter of nodules, the possibility of suspicious nodules detected by imaging as HCC is also increasing [14]. The real-time evaluation of contrast-enhanced ultrasonography in the arterial phase is helpful to analyze the vascular phase characteristics of benign and malignant tumors in detail. On the other hand, the contrast-enhanced pattern of nodules in the portal phase and delayed phase relative to the surrounding hepatic parenchyma (showing continuous enhancement or clearance) is helpful to further distinguish benign from malignant nodules.

Some studies have shown that contrast-enhanced ultrasound can significantly improve the diagnostic accuracy of small hepatocellular carcinoma. The relevant ultrasound parameters provided by CEUS quantitative analysis technology can accurately reflect the microvascular perfusion of tumor lesions. The enhancement of CEUS in HCC is characterized by rapid improvement in arterial phase, enhancement in portal venous phase and delayed phase, and decrease in hypoechoic changes [15]. In this study, the hemodynamic characteristics of patients with stage I-II liver cancer and stage III-IV liver cancer are compared. The results show that the arterial phase was enhanced rapidly in both groups. The blood supply of hepatic artery also plays a dominant role in stage III-IV liver cancer, but the feeding artery is dilated and bent and a large number of contrast agents enter rapidly [16]. Hypoechoic changes mainly occurred in the portal venous phase and delayed phase, and short flow vessels and arteriovenous anastomotic branches could be seen in liver lesions. PTEN gene is located on chromosome 10q23.3 and consists of 9 exons. It encodes a protein of 403 amino acids and has phosphatase activity [17]. PTEN protein can inhibit the occurrence and development of tumor by antagonizing the activity of phosphorylase such as tyrosine kinase.

The results show that after the wild-type PTEN gene was transfected into glioblastoma with abnormal gene, the growth and invasive ability of tumor cells are significantly inhibited, and it was found that it could significantly inhibit the activity of tyrosine kinase FAK in tumor cells. Tg737 gene is a newly discovered HCC tumor suppressor gene. Although the Tg737 gene has been confirmed to play an important role in tumorigenesis, including liver, kidney, and pancreas, the research on how it plays a role in the pathogenesis of HCC is still in its infancy. Studies have shown that there are PTEN point mutations and subsequent inactivation due to gene deletion in a variety of human tumors. For example, a specific PTEN germline mutation has been confirmed in familial melanoma and pancreatic cancer. Recent studies have also shown that aberrant methylation of the PTEN promoter is a major cause, including abnormal methylation of 59 CpG islands in the PTEN promoter region. The expression of PTEN protein in 90 cases of hepatocellular carcinoma and paracancerous tissues was detected by immunohistochemical method [18]. The results show that the positive rates of PTEN in liver cancer tissues and paracancerous tissues are 21.1% and 70.0%, respectively, and the positive rates of PTEN are 17.8% and 75.6%, respectively. At the same time, the results of correlation analysis show that the immunohistochemical scores of PTEN and Tg737 are negatively correlated with WT, which indicated that the higher the expression intensity of PTEN and Tg737, the longer the outflow time of contrast medium, and the slower the regression. The immunohistochemical scores of PTEN and Tg737 are positively correlated with RS, suggesting that the positive expression of PTEN and Tg737 was negatively correlated with the inflow velocity of contrast medium. The inactivation of PTEN and Tg737 genes affects the growth of tumor tissue through a variety of mechanisms, which makes the ultrasonic mode of PTEN and Tg737 positive and negative groups show the characteristics of “fast in and fast out”, the inflow speed is faster, and the low enhancement appears earlier. This leads to the increase of tumor malignancy, the increase of tumor microvessel density, the increase of arteriovenous fistula and hepatic artery blood supply, and the decrease of portal vein blood supply and circulatory overload [19]. Together, these factors lead to faster contrast media inflows and outflows, higher RS, and lower WT. The blood supply of portal vein was dominant in PTEN negative patients, and there are abundant blood sinuses in tumor tissues. The edge of the contrast microbubble is clear, so the inflow speed of the contrast medium is lower and the outflow time is longer.

## 5. Conclusion

Liver cancer is one of the most common malignant tumors in China, with a high incidence in the southeast coastal areas. In conclusion, this study confirmed that conventional ultrasound and liver CEUS can successfully evaluate the expression of PTEN protein in HCC, repeated and noninvasive. Therefore, we know more about the severity of liver cancer and the progress of its prognosis. It is of great significance for the clinical treatment of liver cancer.

## Figures and Tables

**Figure 1:** Ultrasonographic characteristics of liver cancer.

**Figure 2:** Western blot analysis for the expression of PTEN and Tg737 protein.

**Figure 3:** Immunohistochemical detection of PTEN protein in tissues.

**Figure 4:** Immunohistochemical detection of Tg737 protein in tissues.

**Figure 5:** Correlation analysis of immunohistochemical scores of PTEN, Tg737, and RS.

**Figure 6:** Effects of PTEN and Tg737 expression on patient prognosis.

**Table 1:** Correlation between ultrasound characteristics and pathological stage.

Index	I-II stage (*n* = 50)	III-IV stage (*n* = 40)	*χ* ^2^ value	*P* value
Arterial phase			0.725	0.696
High echo	39	34		
Moderate echo	7	4		
Low echo	4	2		
Portal phase			8.706	0.003
High echo	0	0		
Moderate echo	4	13		
Low echo	46	27		
Delay period			0.110	0.740
High echo	0	0		
Moderate echo	4	4		
Low echo	46	36		

**Table 2:** Effects of PTEN expression on the CEUS parameters.

Index	PTEN expression		*t* value	*P* value	Tg737 expression		*t* value	*P* value
	Negative (*n* = 71)	Positive (*n* = 19)			Negative (*n* = 74)	Positive (*n* = 16)		
IMAX	0.92 ± 0.06	0.93 ± 0.08	−0.677	0.500	0.91 ± 0.07	0.94 ± 0.10	−1.432	0.159
mTT	80.7 ± 19.6	81.6 ± 18.5	−0.221	0.825	81.3 ± 18.5	81.9 ± 19.1	−0.116	0.907
TTP	15.9 ± 3.8	16.3 ± 3.5	−0.513	0.609	15.6 ± 3.6	15.9 ± 4.0	−0.296	0.768
RS	16.9 ± 4.5	10.2 ± 3.8	7.512	0.000	17.3 ± 4.8	10.1 ± 4.1	5.570	0.000
WT	19.8 ± 5.4	28.5 ± 4.3	−8.297	0.000	19.7 ± 5.2	29.6 ± 3.7	−7.215	0.000

## Data Availability

The simulation experiment data used to support the findings of this study are available from the corresponding author upon request.
